# Abdominal Computed Tomography Enhanced Image Features under an Automatic Segmentation Algorithm in Identification of Gastric Cancer and Gastric Lymphoma

**DOI:** 10.1155/2022/2259373

**Published:** 2022-07-26

**Authors:** Lihua Zhou, Hao Hu, Lei Zhou, Yi Zhou

**Affiliations:** Department of Radiology, Wuhan Fourth Hospital, Wuhan, 430034 Hubei, China

## Abstract

To analyze the application value of CT-enhanced scanning based on artificial intelligence algorithm in the diagnosis of gastric cancer and gastric lymphoma, the CT images of 80 patients with Borrmann type IV gastric cancer or primary gastric lymphoma diagnosed by endoscopic pathology were retrospectively collected. Meanwhile, a lymph node recognition algorithm based on OTSU threshold segmentation was proposed for CT image processing. The results showed that the missed diagnosis rate of suspected lymph nodes and the missed lymph node detection rate of this algorithm were substantially lower than those of other algorithms (*P* < 0.05). The probability of gastric wall motility disappearance, perigastric fat infiltration, and type A enhancement pattern in the Borrmann type IV gastric cancer group was higher than that in the gastric lymphoma group, with remarkable differences (*P* < 0.05). There was no remarkable difference between the Borrmann type IV gastric cancer group and the gastric lymphoma group in the probability of swollen lymph nodes under the renal hilum (*P* > 0.05). In addition, 5the sensitivity (83.17%), specificity (95.52%), and accuracy (93.08%) of the combined detection of the three CT signs (stomach wall motility, perigastric fat infiltration, and enhancement mode) were substantially improved compared with those of a single sign (*P* < 0.05). To sum up, the lymph node recognition algorithm based on OTSU threshold segmentation had better performance in detecting gastric lymph nodes than traditional algorithms. The CT image characteristics of gastric wall motility, perigastric fat infiltration, and enhancement pattern based on artificial intelligence algorithms were effective indicators for distinguishing gastric cancer and gastric lymphoma.

## 1. Introduction

Gastric cancer is one of the most common gastrointestinal malignancies, ranking among the top five in both morbidity and mortality internationally [1]. Gastric lymphoma is a kind of gastric tumor, originating from the submucosal lymphatic tissue of the stomach, and its incidence ranks second to gastric tumor [2, 3]. The symptoms of gastric lymphoma and gastric cancer are very similar, with abdominal pain, abdominal distension, and abdominal mass being the most common. In addition, some patients do not have abnormal symptoms in the early stage and can only be detected in the physical examination, which largely depends on gastroscopy [4, 5]. Although gastric cancer and gastric lymphoma are similar in pathology, it is easy to cause confusion, which brings great difficulties to the actual identification. However, there are remarkable differences in clinical treatment and prognosis. Therefore, it is still a problem to be studied to find an appropriate detection method to distinguish the two diseases [6, 7].

Imaging technology provides an ideal way for differential diagnosis of gastric cancer and gastric lymphoma, and each imaging method has its own advantages and disadvantages. Fluorodeoxyglucose (18F-FDG) positron emission computed tomography and computed tomography (PET/CT) can simultaneously improve the anatomical and functional data of patients, which is of great help to the early detection of gastric lymphoma. However, the cost of this examination method is relatively expensive, which is beyond the affordable range of ordinary families, and there are false negative diagnoses [8–10]. The low price upper gastrointestinal barium meal can show the softness of the gastric wall and dilation of the gastric cavity as well as gastric mucosa. However, these signs are not specific, and other organs and lymph node metastasis cannot be observed. Endoscopic ultrasonography can detect the extent and depth of gastric wall invasion and find metastatic lymph nodes around the stomach. However, the detection of distant metastasis is also inadequate. Multislice computed tomography (MSCT) has obvious advantages in showing invasion or metastasis of surrounding tissues and organs, as well as abdominal lymph node metastasis, and is the preferred noninvasive examination for gastric tumor staging and surgical feasibility evaluation [11].

With the improvement of people's awareness of physical examination, more and more people go to hospitals for physical examination, and it is increasingly difficult for doctors to evaluate image data manually, resulting in increased work burden [12]. The traditional manual diagnosis method is time-consuming and laborious and easy to misdiagnose and miss diagnosis. It is extremely dependent on the experience and knowledge level of doctors. Therefore, it is necessary to find an intelligent and efficient image data auxiliary analysis method. A computer-aided diagnosis system (CAD) involves digital image enhancement, computer vision, artificial intelligence, and other interdisciplinary fields, which uses advanced mathematical models to analyze and process medical images. Combined with new ideas in the fields of image segmentation, enhancement, and pattern recognition, the diseased areas in medical images can be detected to help doctors understand and diagnose cases more objectively and accurately, which can effectively reduce misdetection and missed detection in clinical diagnosis [13]. For some specific organs, CAD can extract the key information of organs or tissue structure from the photographic image and identify the target in the slice map according to the specific knowledge on the basis of correct segmentation, so as to realize auxiliary detection. OTSU [14], one of the widely used image segmentation methods, is a standard to determine segmentation threshold by calculating the maximum interclass variance or the minimum intraclass variance of image gray level. The specific operation method can traverse all gray levels of digital image gray level histogram as an image gray level segmentation threshold. At each threshold, the image grayscale is divided into two categories according to the threshold value. If, under a certain threshold, the variance between two types of gray values reaches the maximum or the variance within the class reaches the minimum, the threshold is the optimal segmentation threshold.

In summary, the use of the artificial intelligence algorithm to assist doctors in clinical diagnosis is a hot research topic. Therefore, a lymph node recognition algorithm based on OTSU threshold segmentation was constructed in this research. Eighty Borrmann patients with type IV gastric cancer or primary gastric lymphoma were examined in combination with enhanced CT scans. By analyzing the CT image characteristics of the two patients, the application value of enhanced CT scan based on the artificial intelligence algorithm in the diagnosis of gastric cancer and gastric lymphoma was discussed.

## 2. Materials and Methods

### 2.1. Research Objects

In this study, 80 patients from October 15, 2016, to May 20, 2021, who were diagnosed with Borrmann type IV gastric cancer or primary gastric lymphoma by endoscopic pathology were retrospectively enrolled, and their gender, age, height, weight, and CT imaging data were collected. This study had been approved by the ethics committee of the hospital. Informed consent was obtained from patients and their guardians.

Inclusion criteria were as follows: (I) patients with complete clinical data, (II) patients who had signed informed consent, (III) patients older than 20 years, and (IV) patients who had not received treatment. Exclusion criteria were as follows: (I) patients without preoperative enhanced CT scan, (II) patients with poor gastric filling, (III) patients with distant metastasis, and (IV) patients with poor image quality.

### 2.2. CT Scan

All the inspection devices were Philips Ingenuity 64-row 128-slice spiral CT. Patients were scanned in supine position with advanced head and breath-holding mode. The scan was from the tip of the lung to the bottom of the lung. Specific parameters were as follows: tube voltage of 120 KV, intelligent automatic tube current of 150 mA~300 mA, rotation time of 0.75 s/r, pitch of 1.014 : 1, and matrix of 512 × 512. The scanning layer thickness and layer spacing were both 4 mm, and the reconstruction layer thickness was 1 mm.

The enhanced CT images were transferred to the workstation for processing. Related signs were recorded, including peristalsis of the gastric wall, infiltration of perigastric fat, enlarged lymph nodes below hilar level, and enhancement pattern. From the arterial stage to the delayed stage, the thickened gastric wall was strengthened from the inward to the outward through the wall, which was regarded as type A, and the other strengthening methods were regarded as type B. The sensitivity, specificity, and accuracy of the combined detection of three CT signs (gastric wall peristalsis, perigastric fat infiltration, and enhancement mode) were calculated based on the gold standard of endoscopic pathological diagnosis.

### 2.3. Lymph Node Recognition Algorithm Based on OTSU Threshold Segmentation

Clinical observation found that the lymph nodes are mainly located in the fatty tissue around the stomach wall. There is adipose tissue in the inner layer of human skin, and there are no lymph nodes in this part of the adipose tissue. Therefore, the image requires to be preprocessed first. Morphological operations are adopted to perform morphological closing operations on the stomach image to eliminate small cavities in the image, and then, corrosion operations are implemented to remove the strip-shaped examination bed [15].

Dilation is a dual operation of the erosion operation. Under the constraints of structural elements, the background in contact with the target area is merged into the target, so that the target boundary expands outward, and the area of the object increases by a corresponding number of points [16]. It is assumed that the image to be operated is *h*, and there is the following equation.

(1) $$\begin{array}{c} h⊕c=\left\{x\left|\left[{\left(\overset{⟶}{c}\right)}_{x^{\prime }}\cap h\right]\neq \Phi \right.\right\}, \end{array}$$

where *c* represents the structure operator, ⊕ is the operation symbol, and *h* ⊕ *c* is the expansion operation.

The image erosion operation is similar to median smoothing. First, the minimum value in a neighborhood of each position (median smoothing is the middle value) is taken and set as the output pixel value of that position. The neighborhood here is not limited to a rectangular structure but also includes an elliptical structure and a cross-shaped structure. The equation is expressed as follows.

(2) $$\begin{array}{c} h\Theta c=\left\{x\left|c_{x}\subseteq h\right.\right\}. \end{array}$$

The open operation [17] refers to etching first and then expanding, which can eliminate small areas with higher brightness, separate objects at slender points, etc., which is expressed as the following equation.

(3) $$\begin{array}{c} h•c=\left(h\Theta c\right)⊕c. \end{array}$$

*h*•*c* represents the open operation. The closed operation refers to expanding first and then corroding. It has the function of filling small black areas in a white object and connecting adjacent objects. It can also smooth the boundary without changing its area substantially. It is expressed as the following equation.

(4) $$\begin{array}{c} h\circ c=\left(h⊕c\right)\Theta c, \end{array}$$

*h*∘*c* represents closed operation. *h*Θ*c* represents a corrosive operation. After the examination bed is removed, the subcutaneous fat needs to be removed next. First, it is necessary to perform a 4-direction search on the image to find the outermost pixels and then mark the pixel band with a width of 15 pixels within this layer as an area of no interest and remove the human subcutaneous fat layer. The specific steps are shown in Figure 1. The first and last nonzero element positions of each row of the image are searched, and then, the first and last nonzero element positions of each column of the image are searched, so as to obtain the outermost pixel of the image. Then, a 15 × 15 window is fabricated with each outermost pixel as the center. The area outside the window is marked as an area of no interest, which can be eliminated by the morphological operator.  Figure 2 shows the preprocessing results of actual stomach CT images.

The region of interest (ROI) often contains important diagnostic information and, although it may be small in size in the overall image, has a high cost of misrepresentation. Therefore, it is necessary to find a reasonable way to extract the ROI. In gastric CT, grayscale of the liver and lung is evenly distributed without drastic mutation. As the ROI contains a variety of tissue structures, fat, blood vessels, miscellaneous points, and lymph nodes, which exist in it at the same time, the gray levels of the region are substantially different and the gray consistency of the region is poor. Therefore, selecting seed sites in organs is equivalent to selecting seed sites in areas of strong consistency. The gray consistency region and the region of interest can be distinguished by extracting the features that can express the regional gray difference.

Firstly, the consistency region is marked, and a window with a size of 25 × 25 is made with any pixel in the preprocessed image as the center. The features of regional mean and regional variance are then extracted. It is expressed as the following equation.

(5) $$\begin{array}{c} U\left(x_{i}\right)=\overset{m}{\underset{e=1}{\sum }}\frac{l_{e}}{m},\\ \delta \left(x_{i}\right)=\overset{m}{\underset{e=1}{\sum }}{\left[l_{e}-U\left(x_{i}\right)\right]}^{2}. \end{array}$$

*U*(*x*_*i*_) represents the regional average feature, *δ*(*x*_*i*_) represents the regional variance feature, *l*_*e*_ represents the gray value of each pixel in the area where the pixel *x*_*i*_ is located, and *m* represents the number of pixels. After the above characteristics are obtained, a histogram analysis of all variances is performed to obtain a threshold. The area with a variance less than the threshold is marked as a consistent area, and an area with a variance greater than the threshold is marked as a region of interest. Then, the OTSU is used for image binarization segmentation, and the image size is set to *P* × *Q*; then, the following equation is given.

(6) $$\begin{array}{c} p\left(b\right)=\frac{\sum_{h\left(i,j\right)=b}^{\sum }1}{P\times Q}. \end{array}$$

*p*(*b*) represents the frequency of the gray value of *b* and *h*(*i*, *j*) represents the gray value. If there is a gray value *a*, the segmented target area and background area are *h*(*i*, *j*) < = *a* and *h*(*i*, *j*) > *a*, respectively. Then, the proportion of the target part and the number of pixels, the proportion of the background part and the number of pixels, the target mean, the background mean, the total mean, and the interclass variance value can be expressed as the following equations.

(7) $$\begin{array}{c} \varphi_{0}\left(a\right)=\underset{0<i<=a}{\sum }p\left(i\right),\\ M_{0}\left(a\right)=P\times Q\underset{0<i<=a}{\sum }p\left(i\right),\\ \varphi_{1}\left(a\right)=\underset{a<i<=m-1}{\sum }p\left(i\right),\\ M_{1}\left(a\right)=P\times Q\underset{a<i<=m-1}{\sum }p\left(i\right),\\ \kappa_{0}\left(a\right)=\underset{0<i<=a}{\sum }\frac{ip\left(a\right)}{\varphi_{0}\left(a\right)},\\ \kappa_{1}\left(a\right)=\underset{a<i<=m-1}{\sum }\frac{ip\left(a\right)}{\varphi_{1}\left(a\right)},\\ \kappa_{\text{total}}=\varphi_{0}\left(a\right)\cdot \kappa_{0}\left(a\right)+\varphi_{1}\left(a\right)\cdot \kappa_{1}\left(a\right),\\ \varpi =\varphi_{0}\left(a\right)\cdot {\left(\kappa_{0}\left(a\right)-\kappa \right)}^{2}+\varphi_{1}\left(a\right)\cdot {\left(\kappa_{1}\left(a\right)-\kappa \right)}^{2}. \end{array}$$

*φ*_0_ is the proportion of the target part, *M*_0_ is the number of target pixels, *φ*_1_ is the proportion of the background part, *M*_1_ is the number of background pixels, *κ*_0_ is the target mean, *κ*_1_ is the background mean, *κ*_total_ is the total mean, and *ϖ* is the variance between classes.

Then, the image optimal threshold *d* can be expressed as the following equation.

(8) $$\begin{array}{c} d=\underset{0<=i<=m-1}{\text{argmax}}\left[\varphi_{0}\left(a\right)\cdot {\left(\kappa_{0}\left(a\right)-\kappa \right)}^{2}+\varphi_{1}\left(a\right)\cdot {\left(\kappa_{1}\left(a\right)-\kappa \right)}^{2}\right]. \end{array}$$

The OSTU method is used to obtain the theoretical optimal threshold, but in actual operation, the stomach CT image is not simply divided into two but is divided into four regions. Therefore, if the OSTU method is improved and applied to multithreshold segmentation, the multithreshold interclass variance can be expressed as the following equation.

(9) $$\begin{array}{c} \varpi =\overset{m-1}{\underset{j=0}{\sum }}\varphi_{j}\left(a\right){\left(\kappa_{j}\left(a\right)-\kappa \right)}^{2}. \end{array}$$

*φ*_*j*_ represents the pixel ratio of the *j*-th category and *κ*_*j*_ represents the gray value of the *j*-th category. The lymph node recognition algorithm based on regional consistency and OTUS threshold segmentation in this research is marked as RO-OTUS.

### 2.4. Performance Evaluation Indexes

The feasibility of the algorithm in this research is evaluated based on the average omission of the marked suspected lymph nodes and lymph nodes in each case. The missed detection rate of suspected lymph nodes refers to the ratio of the number of suspected lymph nodes missed by the computer to the number of manually labeled lymph nodes, which is expressed as the following equation.

(10) $$\begin{array}{c} \alpha_{i}=\frac{\sum_{j=1}^{L}\alpha_{i,J}}{L}. \end{array}$$

*α*_*i*,*J*_ represents the suspected lymph node missed detection rate of the *j*-th slice of the *i*-th sample, *L* represents the number of all the slices of the *i*-th sample, and *α*_*i*_ represents the average suspected lymph node missed detection rate of the *i*-th sample.

The lymph node missed detection rate is the ratio of the number of lymph nodes missed by the computer to the number of manually labeled lymph nodes, which is expressed as the following equation.

(11) $$\begin{array}{c} \beta_{i}=\frac{\sum_{j=1}^{L}\beta_{i,J}}{L}. \end{array}$$

*β*_*i*,*J*_ represents the missed detection rate of suspected lymph nodes of the *j*-th slice of the *i*-th sample and *β*_*i*_ represents the average missed detection rate of suspected lymph nodes of the *i*-th sample.

In addition, a low-rank model-based suspected lymph node tracking algorithm (LR) [18] and a regional overlap-based suspected lymph node tracking algorithm (RO) [19] are introduced into this article for comparison with the RO-OTUS algorithm.

### 2.5. Statistical Methods

SPSS 19.0 was used for data processing in this study. Mean ± standard deviation ($\bar{x}\pm \text{SD}$) was used for measurement data, and percentage (%) was used for counting data. Pairwise comparison was performed by one-way ANOVA. The difference was statistically remarkable at *P* < 0.05.

## 3. Results

### 3.1. Demographic Variables of Included Patients

In Figure 3, among the 80 patients, 45 were Borrmann type IV gastric cancer patients, 29 were males, and 16 were females. They were with an average age of 55.37 ± 8.73 years, a height of 167.93 ± 13.57 cm, and a weight of 63.17 ± 7.22 cm. There were 35 cases of primary gastric lymphoma, including 22 males and 13 females. The average age was 53.82 ± 10.22 years, the height was 165.08 ± 15.03 cm, and the weight was 59.78 ± 8.18 cm. Among them, the gender ratio, age, height, and weight of the Borrmann type IV gastric cancer group and patients with primary gastric lymphoma were not statistically remarkable (*P* > 0.05).

### 3.2. Detection Performance of Different Algorithms

Figure 4 shows the comparison of the average omissions of suspected lymph nodes and lymph nodes by the three algorithms. The RO-OTUS algorithm's average missed diagnosis rate of suspected lymph nodes was 3.85%, and the average missed diagnosis rate of lymph nodes was 6.17%. The RO-OTUS algorithm's average missed diagnosis rate of suspected lymph nodes was 7.95%, and the average missed diagnosis rate of lymph nodes was 9.55%. The RO algorithm's average missed diagnosis rate of suspected lymph nodes was 9.06%, and the average missed diagnosis rate of lymph nodes was 11.32%. The average missed diagnosis rate of suspected lymph nodes and the average missed diagnosis rate of lymph nodes of the RO-OTUS algorithm were substantially lower than those of the LR algorithm and RO algorithm (*P* < 0.05).

Figure 5 shows the detection results of suspected lymph nodes on gastric CT images by three algorithms. The RO-OTUS algorithm was more comprehensive in the detection of suspected lymph nodes, showing the suspected lymph nodes that were completely infiltrated in the adipose tissue and the suspected lymph nodes that were not completely infiltrated in the adipose tissue.

### 3.3. CT-Enhanced Image Data of Gastric Cancer and Gastric Lymphoma

Figure 6 shows the CT images of a gastric lymphoma (female patient, 67 years old, with epigastric pain for more than 3 months). Routine examination of tumor markers showed 1.6 ng/mL alpha-fetoprotein, 1.2 ng/mL carcinoembryonic antigen, and 65.8 ng/mL ferritin. Gastroscopy pathology was consistent with diffuse large B-cell lymphoma.  Figure 7 shows the CT images of a case of gastric cancer (patient female, 45 years old). The chief complaint was malignant vomiting for half a year. The vomitus was gastric contents, which can be diagnosed as gastric horn ulcer-type well-differentiated adenocarcinoma.

### 3.4. Comparison of CT Signs of Gastric Cancer and Gastric Lymphoma

In Figure 8, Borrmann type IV gastric cancer and primary gastric lymphoma had remarkable differences in gastric wall motility, perigastric fat infiltration, and enhancement patterns (*P* < 0.05). There was no notable difference in enlarged lymph nodes under the renal hilum (*P* > 0.05).

### 3.5. Joint Detection Performance of CT Signs

In Figure 9, the sensitivity (83.17%), specificity (95.52%), and accuracy (93.08%) of the joint detection of the three CT signs (stomach wall motility, perigastric fat infiltration, and enhancement mode) were substantially improved compared with those of a single sign (*P* < 0.05).

## 4. Discussion

Gastric cancer and primary gastric lymphoma are the two most common malignant tumors in the stomach, but the accurate distinction between the two is of great significance because of the difference in clinical treatment mode and prognosis [20]. Endoscopy is the gold standard for early diagnosis of gastric disease, but it is prone to missed diagnosis and misdiagnosis. In addition, gastric cancer and primary gastric lymphoma show similar images on the image, which will lead to greater obstacles to the physician's subjective judgment. It is urgent to find an intelligent detection method to assist physicians in clinical diagnosis [21, 22]. In this research, the lymph node recognition algorithm based on OTSU threshold segmentation was constructed, and its performance was analyzed. The results suggested that the average missed diagnosis rate of suspected lymph nodes and the average missed diagnosis rate of lymph nodes of the RO-OTUS algorithm were substantially lower than those of the LR algorithm and the RO algorithm (*P* < 0.05), which was similar to the findings of Findlay et al. [23]. It showed that the RO-OTUS algorithm constructed can improve the diagnostic accuracy of CT-enhanced images and had clinical promotion value. Judging from the detection results of suspected lymph nodes in gastric CT images, the RO-OTUS algorithm was relatively more comprehensive in detecting suspected lymph nodes. The suspected lymph nodes that were completely infiltrated in the adipose tissue and the suspected lymph nodes that were not completely infiltrated in the adipose tissue were shown, which corresponded to the results of the above quantitative data.

The CT images of 80 patients with Borrmann type IV gastric cancer or primary gastric lymphoma diagnosed by endoscopic pathology were retrospectively collected and analyzed. The CT signs of gastric cancer and gastric lymphoma were compared, and it was found that Borrmann type IV gastric cancer and primary gastric lymphoma had remarkable differences in gastric wall motility (*P* < 0.05). The reason may be that the lymphoma cells of lymphoma mainly infiltrate and grow, and normal gastric parietal cells are generally not damaged and still have a certain degree of expandability and flexibility. Borrmann type IV gastric cancer has diffuse infiltration of the gastric wall, and normal gastric wall tissue is destroyed, causing necrosis and fibrosis inflammatory reaction and ultimately leading to the destruction of the gastric wall and stiffness [24]. In addition, there was a remarkable difference between Borrmann type IV gastric cancer and primary gastric lymphoma in perigastric fat infiltration (*P* < 0.05). This was consistent with results of Hölscher and Law [25] who proposed that the probability of perigastric fat space infiltration in primary gastric lymphoma was lower than that in gastric cancer, which suggested that perigastric fat space infiltration could be used as an indicator to judge gastric cancer and primary gastric lymphoma. Borrmann type IV gastric cancer and primary gastric lymphoma had remarkable differences in the enhancement mode (*P* < 0.05). This phenomenon can be explained by the histopathological composition of the two. The capillaries in the mucosal layer of gastric cancer are very rich, and the blood supply is obvious, so the arterial phase begins to strengthen, and the venous phase and the delayed phase still have a large amount of contrast agent retained in the tortuous and deformed tumor blood vessels, showing delayed enhancement [26]. There was no statistically remarkable difference between Borrmann type IV gastric cancer and primary gastric lymphoma in terms of enlarged lymph nodes under the renal hilum (*P* > 0.05). Although the size of the lymph node is often used to determine whether the lymph node has metastasized before surgery, there is no uniform standard for the diameter threshold used to determine the metastasis of the lymph node, and it is not uncommon for cancer cells to be found in normal-sized lymph nodes. Therefore, this result is in line with clinical routine cognition [27]. The performance analysis of the combined detection of CT signs found that the sensitivity (83.17%), specificity (95.52%), and accuracy (93.08%) of the joint detection of the three CT signs (stomach wall motility, perigastric fat infiltration, and enhancement mode) were substantially improved compared with those of a single sign (*P* < 0.05). This indicated that the joint detection of gastric wall motility, perigastric fat infiltration, and enhanced mode can improve the accuracy of identification of gastric cancer and gastric lymphoma.

## 5. Conclusion

In this study, 80 patients who were diagnosed with Borrmann type IV gastric cancer or primary gastric lymphoma by endoscopic pathology were retrospectively enrolled, and their gender, age, height, weight, and CT imaging data were collected. The results showed that the enhanced CT images based on an automatic segmentation algorithm could clearly display the imaging features of gastric cancer and primary gastric lymphoma. Moreover, joint detection of gastric wall peristalsis, perigastric fat infiltration, and enhancement pattern on CT can improve the clinical differential accuracy of gastric cancer and gastric lymphoma. However, this research lacks multicenter external validation experiments and does not analyze the consistency between subjective signs and evaluators of image omics features. Patient sample data will continue to be collected in the future to further analyze the clinical application value of the artificial intelligence algorithm combined with CT images. In conclusion, this study provides data support for the differential diagnosis of gastric cancer and primary gastric lymphoma.

## Figures and Tables

**Figure 1:** Image preprocessing process.

**Figure 2:** Display of preprocessing results of stomach CT images: (a) original image; (b) image of the examination bed removed; (c) image of the subcutaneous fat removed.

**Figure 3:** Patients' demographic variables: (1) Borrmann type IV gastric cancer and (2) primary gastric lymphoma. (a) Gender ratio and age and (b) weight and height.

**Figure 4:** Comparison of the average omissions of suspected lymph nodes and lymph nodes by the three algorithms. ^∗^Compared with the proposed algorithm (*P* < 0.05).

**Figure 5:** The detection results of three algorithms for suspected lymph nodes in gastric CT images. Blue indicated suspected lymph nodes: (a) original image; (b) RO-OTUS algorithm; (c) LR algorithm; (d) RO algorithm.

**Figure 6:** CT images of lymphoma (female patient, 67 years old).

**Figure 7:** CT images of gastric cancer (female patient, 45 years old).

**Figure 8:** Comparison of CT signs of gastric cancer and gastric lymphoma. (A) Borrmann type IV gastric cancer and (B) primary gastric lymphoma. ^∗^There was a remarkable difference between Borrmann type IV gastric cancer and primary gastric lymphoma (*P* < 0.05).

**Figure 9:** Joint detection performance of CT signs. a: gastric wall motility; b: gastric fat infiltration; and c: enhanced mode. (a) Detection performance of a, b, and c. (b) Joint detection performance of a+b, a+c, and b+c. (c) Joint detection performance of a+b+c.

## Data Availability

The data used to support the findings of this study are available from the corresponding author upon request.
